# The Generation and Realization of Dunhuang Cultural Values from the Perspective of Crosscultural Communication: Based on Spanish and Chinese Culture

**DOI:** 10.1155/2022/5382213

**Published:** 2022-10-03

**Authors:** Lin Liang, Shasha Wang

**Affiliations:** ^1^Center for Bilingual Lexicography and Bilingual & Bicultural Studies, Xiamen University, Fujian, Xiamen 361005, China; ^2^Translation and International Studies Department, Universidad Autónoma de Barcelona, 08193, Spain

## Abstract

Dunhuang Feitian is a complex of Indian culture, Buddhist culture, Western culture, and Central Plains culture. It has been loved by artists since ancient times and is an important embodiment of the essence of grotto art. Dunhuang culture is an important cultural heritage used to build Chinese cultural identity. With the development of science and technology and the progress of society, the exchanges between cultures are increasingly deepened. These exchanges are not only reflected in language, economy, politics, film, and technology but also in science and technology. From a macroperspective, culture includes all products, and products are also an intuitive manifestation of culture. How to continue culture and consider the customs and taboos of the outside world while continuing retains the essence of culture to the greatest extent and integrates local characteristics, so that foreign culture can be integrated into it. Being well accepted by local people will become an important proposition for crosscultural communication and value expression. Therefore, based on cognitive thinking and Kansei engineering theory, this research explores and analyzes product design methods that integrate Spanish and Chinese cultures, hereinafter referred to as “Western-Chinese” cultures. Analyze the two cultures separately: from a certain culture, after the image investigation, extract the target image; from another culture, get the modeling design factors and then realize the product image modeling design of crosscultural Dunhuang integration and the Dunhuang culture. Value generation and realization reasonably recognize the connection between the two cultures, form a crosscultural integration design theory, and provide new ideas for product innovation design.

## 1. Introduction

Located at the western end of the Hexi Corridor, Dunhuang was an important fortress on the ancient Silk Road. Dunhuang, the Eastern Han scholar Ying Shao, explained it as “ Dun , Daye, Huang, Shengye.” It was the barrier for the Central Plains Dynasty to rule the Western Regions, and it was also the center of the cultural exchange between the Central Plains and the Western Regions. During the Han Dynasty, Buddhism was introduced to China via the “Silk Road,” and Dunhuang was the only place where Buddhism spread eastward. During the nearly thousand years of development from the Han Dynasty to the Tang Dynasty, Buddhist culture gradually improved its own connotation and local style after experiencing the conflict and fusion with traditional Chinese culture. Dunhuang culture is very historical and artistic, especially the Dunhuang Mogao Grottoes, which are admired by the world, are the artistic treasures left by Dunhuang Buddhism to the world, and more than 90% of the precious Tibetan scripture cave documents are Buddhist books. From these grotto murals and Buddhist scriptures, we can all feel the splendid development of Buddhist culture in Dunhuang at that time. Cultures vary from country to country, and in the context of increasing globalization, the exchange between cultures is indispensable. The study of Dunhuang culture is an important branch of Dunhuang studies. At the same time, the glorious period of Dunhuang cultural development is the period from the Han Dynasty to the Tang Dynasty, and this period is also the most creative and inclusive stage of the entire Chinese culture. The splendor of Dunhuang culture is the epitome of the prosperity of the Han and Tang dynasties. Learning the splendid culture left to us by these ancestors can inspire our patriotism and national cultural confidence and also remind us to better inherit the Chinese civilization. Since the end of the nineteenth century, academic circles at home and abroad have made valuable explorations of Dunhuang culture. Professor Hao Chunwen, a well-known scholar of Dunhuang studies, once said that after entering the 21st century, the development of Dunhuang studies is no longer just about pursuing new material content but also combining with other disciplines, exploring new methods, and thinking about new issues. Different from traditional Dunhuang cultural studies, from the perspective of crosscultural and value realization, the organic combination of Dunhuang culture and different cultures is the guarantee for the vitality and progress of Dunhuang studies. In the late 1980s, domestic research on “cross-cultural” started, and today, “cross-cultural” research has achieved certain results in various aspects, such as crosscultural communication, crosscultural management, and crosscultural advertising aspect. With the development of the times, the study of cultural differences will also be integrated into product design, and “cross-culture” will also be studied as an entry point for modern design [1–9].

This study selects the Dunhuang culture in the Han and Tang dynasties as the research object. As a very successful case of crosscultural communication, Dunhuang culture obviously has a very high crosscultural research value. This research takes the design of crosswestern and Chinese cultural products as the research theme, analyzes the imagery and design factors of the two cultures, and studies the user's cognition in the extraction process, so as to provide reference for contemporary globalized crosscultural product design. At the same time, it also reflects the value of Dunhuang culture from the side.

## 2. Related Work

During the Sui and Tang dynasties, the society was in a stage of rapid development. Dunhuang, which is connected with China and foreign countries, became a prosperous international metropolis at that time. The prosperous environment made the multiethnic and diversified social characteristics developed to the extreme at that time. The process of ethnic fusion and cultural integration continued to evolve in Dunhuang and gradually developed into a situation in which the Central Plains Confucian culture was the main body and the cultures of various ethnic groups coexisted. This prosperous scene is the core of multiethnic cultural exchanges in the Hexi Corridor of the prosperous Tang Dynasty feature. During the Five Dynasties period, Dunhuang was a time of division and turmoil. Political rights were frequently replaced, and the phenomenon of division and division continued to occur. At this time, Dunhuang experienced successively being ruled by Tubo, Guiyi Army, Jinshan Kingdom, and Cao's regime. During this process, the phenomenon of clashes and mutual integration between cultures also persisted. The rulers of Xixia have Buddhist beliefs and attach great importance to economic development. So far, there are still a lot of Buddhist art in the Mogao Grottoes. The development of Dunhuang in the Yuan Dynasty gradually withered away. The Ming Dynasty attached great importance to the role of waterways, the Silk Road was abandoned, and Jiayuguan Pass was closed. Since then, Dunhuang has been unorganized for nearly two hundred years, and the development of the Dunhuang area has been resumed since the Qing Dynasty. In 1900, Taoist priest Wang Yuanlu accidentally discovered the cave, which attracted foreign explorers to Dunhuang to hunt for treasures. Since then, Dunhuang literature has been scattered all over the world. To sum up, the evolution and development of Dunhuang culture are a process of multicultural and multiethnic exchanges and mutual integration and finally evolved into a mode dominated by the Central Plains culture and compatible with various cultural characteristics. The process of crossinfluence of different cultures in this area has made the structure of Dunhuang culture more diverse, open, contemporary, and inclusive, until it develops into a regional cultural tradition. This kind of temperament of accommodating atmosphere is the basis for cultural mutual learning and exchange and integration in the Hexi Corridor since ancient times. Even today, throughout China, cultural exchanges and mutual learning of various ethnic groups are still taking place and new forms of communication that incorporate the characteristics of the current era. The cultural characteristics of harmony, tolerance, and harmony that have been deposited in my country's cultural genes for thousands of years have become the inexhaustible nourishment for building a new type of ethnic relationship [10–15].

In the process of crosscultural communication with Western countries, the cultural backgrounds of the two parties may be similar or far from each other. People living in different cultural backgrounds have natural ideas, ways of thinking, lifestyles or personality characteristics, etc. For this aspect, the process of crosscultural communication can be understood as “information exchange activities carried out by groups with different historical and cultural characteristics, and at the same time including different cultural elements in various countries and regions. The process of communication and the effect of this activity on global human beings”; second, the encoding and decoding of information are transmitted by individuals or groups from different contexts. It is one of the tools to measure crosscultural communication; thirdly, because of the differences in the semiotic systems of the two parties involved in the communication, crosscultural communication has thus become a process of symbol exchange. This orientation points out the core element of crosscultural communication, that is, the construction of a common meaning space for both parties through different language symbols. In addition to the above three representative aspects of academia, in today's society, the analysis of crosscultural communication needs to consider a new background. At present, the mode of information dissemination has been innovated to a great extent all over the world. The rise of immigrants, the rise and fall of refugee waves, the continuous development of urbanization, etc., have all had a great impact on the global social culture. In terms of cultural dissemination, different countries show an unequal integration phenomenon, and they cannot identify with each other, resulting in friction and contradiction between different cultures, which makes crosscultural communication more and more urgent.

## 3. The Excavation of Dunhuang Cultural Gene and Value between Western and Chinese Cultures

### 3.1. Excavation Methods of Crosscultural Goal Intentions in the West and China

Different cultures have formed unique cognitive symbols due to different factors such as value orientation, historical tradition, and living environment. After a long period of precipitation and accumulation, this simple symbol has become a common historical memory and life emotion shared by people. This kind of symbol is usually a representative thing recognized by people, the spirit of the symbol is extracted from its complicated form, and it is simplified and expressed. These formal symbols are not unique phenomena of individuals but the emotional memory of the common psychology. Cultural symbols are generated in a certain time and space and have greater stability. For example, the word phoenix has formed a unique cultural symbol. In ancient China, it heralded the noble status of women: the so-called “hundred birds facing the phoenix” and “auspicious dragon and phoenix” over understanding. Through a large amount of research and study, the cultural imagery is collected through books, the Internet, newspapers, and interviews with relevant scholars and other means, and the perceptual imagery vocabulary with high frequency is sorted out. These imagery vocabulary can represent the characteristics of the culture. Its specific flow chart is shown in Figure 1 [16].

### 3.2. The Cognitive Way of Dunhuang Cultural Image in the Crosscultural Area of Western and Central China

User cognition can be regarded as a process of information processing and communication. Users receive information from the external environment through their senses for internal processing, so as to recognize things. Cognitive thinking is the process of collecting the information elements produced by people's observation, analysis, and inference of the things being recognized. In the cognitive process, vision is usually the earliest sensory system to discriminate in the cognitive thinking process. Since users ‘identification with crosscultural products mainly comes from visual perception, designers should take the initiative to maintain basically consistent perception information with users visually. In the process of crosscultural product design, it is not only limited to the shaping of crosscultural products by designers but also requires the approval of users, so that the crosscultural products created in this way can stimulate the approval of users. To select the design factors of another culture based on cultural imagery, the expression of images is often the most intuitive. Image Kanban and image scale diagrams are more commonly used expressions. They can convey design concepts well. Therefore, image Kanban is used to eliminate users: the method of image difference. Due to people's cognitive differences, different people perceive the same thing differently. Therefore, it is necessary to use image Kanban to eliminate cognitive differences as much as possible. Through the image Kanban, the matching of cultural target imagery with another cultural design factor can be achieved. The research process is shown in Figure 2. The first is the collection of target image data (images), then the effective images are obtained through the screening of designers, and finally, the image board is established.

### 3.3. Excavation of the Value of the Crosscultural Gene Bank in the West and China

From the concept of crosscultural genes to the exploration of crosscultural genes, the main purpose is to find another cultural designable factor that conforms to the image of crosscultural goals. The research process is shown in Figure 3. Analyze crosscultural genes by using structural models; read the dominant factors in crosscultures and generate crosscultural gene pools; then summarize the dominant factors of the fusion culture by analyzing the map; the design factors that conform to the crosscultural target image are matched and selected to determine the cultural design factors.

#### 3.3.1. The Reading of Crosscultural Genes in Western and Chinese

The hierarchical structure model is an effective method for reading the specific characteristic elements of cultural genes of different countries. For different components, different levels of aggregation and combination are carried out according to the interrelated influence and affiliation between factors to form a multilevel analysis structure model. Genes are viewed as extracting “internal and external” features of a design object. According to the internal characteristics of genes, they are divided into dominant factors and recessive factors. Those that are recognized on the surface are called dominant factors. In crosscultural product design, they generally refer to shapes, colors, patterns, and materials. For the division of genes, the hierarchical structure model is used to deconstruct and stratify cultural genes, as shown in Figure 4 [17]. According to the characteristics of cultural genes, the target objects are selected and divided into dominant factors, which are defined as first-level layers, and then the first-level layers are divided one by one until each factor is figuratively divided.

#### 3.3.2. The Establishment of a Crosscultural Gene Bank between the West and China

Kristofer Schipper first proposed the concept of cultural gene bank in “The Chinese Cultural Gene Bank.” Cultural genes are the basic elements that determine the process of cultural inheritance, and their types are complex and abstract. Then, the establishment of a crosscultural gene bank is not only an important means to improve cultural taste and protect cultural elements but also help to analyze the composition of culture as a whole. Excavation and research on the dominant factors across cultures are carried out, as shown in Figure 5. The data are organized in an orderly arrangement, combination, classification, and hierarchical deconstruction according to the attributes of cultural genes and their internal logical relationships, forming a comprehensive system that can record multiple cultural information. The document library of order is divided into three categories: shape factor library, pattern factor library, and color factor library [18, 19].

Color is not only a feeling but also a kind of information, and it is also one of the important elements for designers to express products. It conveys cultural information and expresses their feelings through vision and is one of the important elements of cultural genes. The main function of color is to symbolize, and a color often has its own fixed meaning. Different colors can affect people's emotions, temperaments, and actions, such as red symbolizing enthusiasm and blue symbolizing indifference, which are the emotional expressions of different colors. In product design, designers use reasonable colors to give users a certain sense of orientation.

Pattern is a predesign of form, color, and structure in practical art, decorative art, and architectural art. A general term for schemes such as patterns and decorative patterns that are made under the constraints of process materials uses economy, production, and other conditions. It reflects the specific cultural connotation through its different shapes, and the pattern is the most typical dominant factor of the pattern. In my country, traditional patterns have a long history and are an important part of our traditional culture, which can most intuitively reflect culture.

Modeling is as follows: the image of the object created is also called modeling. The external modeling refers to “the appearance of an object or figure presented by the combination of external surfaces or lines.” In product design, it refers to the external contour, such as the appearance of a cast object, molds, and patterns. But for culture, it is also one of the important manifestations.

## 4. The Realization of the Value of Dunhuang Cultural Products across Cultures between the West and China

### 4.1. The Form of Dunhuang Cultural Value Conversion between Western and Chinese Cultures

The textual representation of crosscultural values of the design language system is used to formulate plans, standards, and specifications for all levels of the brand in the form of manuals, including the specifications that must be strictly implemented and the recommended specifications that can be used for reference. The Dunhuang crossultural language manual contains three major sections, namely, the brand building level, the design specification level, and the design product display (see Figure 6). The brand level includes brand vision, mission and theme, proposition and brand promise, brand positioning, brand structure, SWOT analysis, user positioning, user needs, and combination parts (product structure division). The brand building level determines the positioning of the superstructure of the brand, which is the core of the brand, and is used to guide all product development behaviors and other corporate behaviors of the brand.

As mentioned above, the crosscultural brand building level includes nine parts: the first is the brand vision. The brand vision is the embodiment of the core values of Dunhuang crosscultural brand and guides the general direction of the development of the entire brand. The public can learn about the brand through the brand vision. Culture finds the point of convergence between oneself and the brand, and the brand vision is “transmitting the meaning of Dunhuang's artistic beauty”; the second is the mission and purpose, and this part is to set the brand mission, so as to guide all the direction of the brand's BI behavior. The mission and purpose of the brand are implemented in each process to achieve the goal of accurately conveying the brand vision; the third is the proposition and brand commitment, which stipulates the brand's detailed commitment and proposition to the public and society, which will be used in subsequent product development and corporate behavior. It is necessary to implement the brand promise; the fourth is the core value and quality, and this part outputs the core values of the brand and the corresponding core quality; the remaining parts are brand positioning, brand structure, SWOT analysis, user positioning, user needs, and combination part (product structure division), and these parts are based on the research on Dunhuang culture and the needs of the audience, determine the direction of brand product development, and establish brand positioning and product design image positioning by importing models and methods constructed by design language [20–23].

The design level in the crosscultural language manual includes design language, brand value and design style observation, logo and its specifications, brand basic graphics, brand and product color, product material, and product shape (shape). The crosscultural design level focuses on the specific specifications of product design and makes corresponding basic standards and usage specifications for the VI and DI parts of the brand. The design level includes the above seven parts. The first is design language: this part explains the relationship between design language and design innovation and constraint norms and shows the necessity of introducing Dunhuang crosscultural brand into the construction of design language system; the second is the observation of brand value and design style: this part mainly defines the brand design style is introduced, the method of semantic cloud analysis in the construction of design language is introduced, and the corresponding transformation of Dunhuang cultural value and brand value is carried out; the third is the brand logo, which is based on Dunhuang mural elements to create a brand that conforms to the Dunhuang style positioning, LOGO, and make a series of standard requirements for the use of brand LOGO; the fourth is the basic graphics of the brand, which is the basic pattern derived from the brand logo, which is used in the design and development of brand products and brand VI design; the fifth is the brand and product color: this part establishes the brand's main color and brand auxiliary color and makes a series of brand and product color reference specifications to provide reference for the design and development of brand products and the establishment of VI visual system colors; the sixth is product material: this part is the reference of some materials for product development; the seventh is the product shape (shape), which is the specific presentation of the design scheme.

### 4.2. Crosscultural Dunhuang Cultural Product Design Product Value Conversion

Based on the guidance planning and design plan of the crosscultural language manual, the textile design and development are carried out with the theme of flying elements, which are divided into two series: traditional direction and modern abstract direction. The traditional directional pattern follows the composition form of the caisson in the grottoes and adopts a diagonally symmetrical composition. It corresponds to the product style positioning analysis in the crosscultural language manual. The traditional pattern is retained, appropriate color adjustment is selected on the color matching specification, and the classic pattern is made by recoloring the traditional elements. The visual presentation is more modern, youthful, and fashionable. The design plan incorporates brand LOGO, extended brand basic patterns, and standard words. The combination of basic patterns and the placement of standard words are strictly in accordance with the LOGO combination part of the crosscultural language manual. The role of the crosscultural language system in the development of crosscultural product series is shown through standard colors, basic brand patterns, and standard brand characters. The details are shown in Figures 7–11.

The modern abstract direction pattern design adopts an abstract composition, which is full of deconstruction and more in line with the modern aesthetic style. Trying to redeconstruct Dunhuang Feitian IP design elements, transform them into very modern DI design elements and integrate abstract composition methods, so that the entire design scheme presents the trend of modernization, personalization, and fashion. Optimize the color scheme based on the color matching reference in the color specification section of the crosscultural language specification manual and integrate the brand LOGO, the extended brand basic pattern, and standard words, and the combination of the basic pattern and the standard word placement is strictly in accordance with the LOGO combination section in the crosscultural language manual to make sure the role of design language in crosscultural product development is shown through standard colors, the use of brand basic patterns, and brand standard words [24], as is shown in Figures 12–15.

The abovementioned crosscultural product design and development practice introduce the tools and methods of design language system construction into the product development process and draw three conclusions based on the whole-process design and development practice: first, the introduction of the design language system stipulates some basic design problems, greatly reducing ineffective design attempts and improving the work efficiency of designers; second, the introduction of the design language system clearly shows the unifying elements of the brand on the product and enhances the brand's sense of series and family in visual effects, so that the brand has the inheritance of the family DNA; third, the success of Dunhuang crosscultural product design and development based on the introduction of the design language system shows the correctness of the decision-making at the brand strategic level, and it is necessary for crosscultural brands to introduce standardization and professional design management method.

### 4.3. Crosscultural Dunhuang Cultural Product Design Product Value Realization

The crosscultural language manual is the product of the method of building the brand introduction system, which has the characteristics of both methods and tools. Its construction process is based on certain steps and models, which play a theoretical role in the construction of crosscultural brands. The crosscultural language manual can guide the construction of brands from 0 to 1 and establish certain standards for the design elements of DI products for the entire brand. At the same time, it also involves the VI part of the brand vision and the MI concept, which is similar to the enterprise CIS system but different from the CIS system. It is a method construction focusing on the design strategy and design leadership. The introduction of design language can help improve the brand strategy system for brands that have not yet started and brands that have just started. In terms of the characteristics of the tool, it refers to the practical significance of the crosscultural language manual for the Dunhuang crosscultural brand. As mentioned above, the crosscultural language manual establishes certain standards and norms about the brand, these standards are presented in the form of the manual, and the manual becomes a branding tool at this time. First, it can limit the unreasonable creative behavior of designers to a certain extent and guide designers to spread their creativity in a reasonable direction. In this process, it can improve the efficiency of designers' work and avoid unnecessary design behaviors; second, the product series developed based on the crosscultural language manual must have strong brand DNA design elements. It can establish a clear and unified brand name card for the enterprise that conforms to the brand culture, can enhance the overall image of the brand, create a sense of quality, and attract consumers at the same time. While increasing revenue for the brand, it successfully transformed the Dunhuang cultural IP into modern factors with the characteristics of the times for dissemination and played a role in the core value of continuing to spread and promote Dunhuang culture in the contemporary era.

## 5. Conclusion

This research starts from the concept of crosscultural integration, applies the theory of Kansei engineering, reasonably selects the design factors of another culture based on the image of one culture, and uses the image board to eliminate the cognitive differences of users, so as to solve the problem of crosscultural integration in product design. Taking the development and design of Dunhuang cultural products as an example, the crosscultural product image modeling design is carried out, which verifies the effectiveness of the method proposed in this study. First of all, sum up the development of Dunhuang culture and Buddhist culture in China, as well as the characteristics and categories of Dunhuang grotto art, summarize the true value of Dunhuang culture by deeply excavating the connotation and significance of Dunhuang culture, and inherit this value to Dunhuang cultural creative brand as a theoretical basis to guide the construction of Dunhuang's crosscultural brand. Secondly, in the subsequent construction of the brand design language system, it guides the positioning of the superstructure of the brand, such as brand positioning, brand cultural connotation, and core value. By intervening in the design language method in the category of design management, it can achieve the development of family and series of Dunhuang cultural and creative brand products. To help cultural and creative brands enhance brand sense and brand value, carry out brand communication more systematically and enhance user loyalty. Finally, it has been proved by practice that the development of brand series products after the intervention of the design language guidance method has effectively improved the design efficiency. In terms of product results, the product series developed by the intervention design language method is obviously more visually unified and attractive and more unified with the brand DNA.

## Figures and Tables

**Figure 1:** Flow chart of target intent mining.

**Figure 2:** Intentional cognition flow chart.

**Figure 3:** Flowchart of crosscultural factors.

**Figure 4:** Crosscultural structure model diagram.

**Figure 5:** West-China crosscultural gene bank.

**Figure 6:** Catalogue of crosscultural language manuals.

**Figure 7:** Feitian series textile pattern design line draft.

**Figure 8:** Color draft of Feitian series textile pattern design.

**Figure 9:** Feitian series textile pattern design-traditional direction circular color draft.

**Figure 10:** Textile pattern design of Feitian series-rectangular color draft in traditional direction.

**Figure 11:** Textile pattern design of Feitian series-schematic diagram of traditional direction element transformation.

**Figure 12:** Feitian series pattern abstract modern direction square color draft.

**Figure 13:** Feitian series pattern abstract modern direction circular color draft.

**Figure 14:** Textile pattern design of Feitian series-a schematic diagram of the transformation of abstract modern directional elements.

**Figure 15:** Product design display.

## Data Availability

The dataset can be accessed upon request.
